This article has been retracted.

# Cell Division Cycle-Associated Protein 3 (CDCA3) Is a Potential Biomarker for Clinical Prognosis and Immunotherapy in Pan-Cancer

**DOI:** 10.1155/2022/4632453

**Published:** 2022-08-30

**Authors:** Yingkun Xu, Meiying Shen, Yang Peng, Li Liu, Lingfeng Tang, Ting Yang, Dongyao Pu, Wenhao Tan, Wenjie Zhang, Shengchun Liu

**Affiliations:** ^1^Department of Breast and Thyroid Surgery, The First Affiliated Hospital of Chongqing Medical University, Chongqing 400042, China; ^2^Department of Breast and Thyroid Surgery, Women and Children's Hospital of Chongqing Medical University, Chongqing 401120, China

## Abstract

CDCA3 is an essential regulator in cell mitosis and can regulate many physiological and pathological processes in the human body by stimulating certain proteins such as cell cycle regulatory proteins, transcription factors, and signal transduction molecules. Although several studies have shown that dysregulation of CDCA3 is a common phenomenon in human cancers, no systematic pan-cancer analysis has been performed. In this study, we comprehensively investigated the role of CDCA3 in 33 human cancer types by utilizing multiple cancer-related databases and bioinformatics analysis tools, including TCGA, GTEx, GEPIA, TIMER, STRING, Metascape, and Cytoscape. Evidence from bioinformatics databases shows that CDCA3 is overexpressed in almost all human cancer types, and its overexpression is significantly associated with survival in patients with more than ten cancer types. CDCA3 expression positively correlates with immune cell infiltration levels in multiple human cancer types. Furthermore, the results of the GSEA analysis revealed that overexpression of CDCA3 may promote the malignant progression of cancer by activating various oncogenic signaling pathways in human cancers. In conclusion, our pan-cancer analysis provides a comprehensive overview of the oncogenic role of CDCA3 in multiple human cancer types, suggesting that CDCA3 may serve as a potential therapeutic target and prognostic biomarker in multiple human cancer types.

## 1. Introduction

With the changes in the disease spectrum, cancer has become a major threat and challenge to human health, and morbidity and mortality have increased yearly, bringing a heavy burden to global public health [1–3]. Worldwide, more than 28.4 million new cancer cases will occur by 2040, a 47 percent increase from 2020 [4]. Early diagnosis and treatment of cancer patients are the most important means to improve the cure rate and survival rate of cancer patients. Compared with pathological biopsy, in early cancer screening, cancer markers have the advantages of noninvasiveness, low cost, convenience, and speed. At the same time, the presence of quantitative changes in cancer markers can indicate the nature of cancer, understand the occurrence, cell differentiation, and function of cancer, and play a vital role in the diagnosis, classification, prognosis, recurrence, and treatment of cancer. As research progresses, researchers have discovered that cancer is a complex genomic disease with multiple forms depending on its location and cellular origin [5]. Although emerging therapies and various targeted drugs are developed for cancer treatment, cancer cannot be cured entirely. Therefore, there is an urgent need to discover early diagnostic tools, predictive biomarkers, and more reliable treatments to improve cancer patients' cure and survival rates [6–10]. The significance of pan-cancer research is to apply diagnosis and treatment to more cancers through cross-cancer similarity [11, 12]. Therefore, identifying cancer markers between different cancer types is helpful for cancer diagnosis and treatment.

Abnormal regulation of cell cycle will lead to uncontrolled excessive proliferation of cells and promote the formation of cancer, which is of great significance in the occurrence and development of cancer. Therefore, the study of cell cycle regulation-related factors is of great significance for revealing the occurrence and development of cancer. The expression of cell division-regulating genes is required in different cell cycle phases. Previous studies have also reported the relationship between cell-cycle regulation-related genes and carcinogenesis [13–15]. With the continuous development and progress of clinical molecular biology, it has been found that cell division cycle-associated protein 3 (CDCA3) is abnormally highly expressed in non-small-cell lung cancer, gastric cancer, bladder cancer, leukemia, colon cancer, and breast cancer [16–21]. CDCA3-encoded protein triggers cell entry into mitosis and is required to properly activate cyclin-dependent kinase 1/cyclin B and cell entry into mitosis [22–24]. In addition, CDCA3 can affect cell cycle progression by affecting DNA methylation [25].

Although more and more pieces of literature report that CDCA3 plays this critical biological role in cancer progression, there is currently a lack of a study that provides a pan-cancer analysis of CDCA3 from a holistic perspective. Therefore, based on TCGA, GTEx, GEPIA, STRING, TIMER, Metascape, and other databases, this study conducted a pan-cancer analysis of CDCA3 in terms of gene expression, prognostic significance, immune correlation, tumor mutation burden, and microsatellites. We hope this study will help cancer researchers deepen their understanding of CDCA3 in pan-cancer.

## 2. Materials and Methods

### 2.1. Data Collection and Processing

In this study, we obtained RNAseq data and corresponding clinical information for all cancer types through The Cancer Genome Atlas (TCGA) database (https://portal.gdc.com). In addition, to increase the data of normal tissue samples, we also obtained RNAseq data of more clinical samples through Genotype-Tissue Expression (GTEx) database (https://gtexportal.org/home/). We analyzed differences in CDCA3 mRNA expression between cancerous and corresponding noncancerous tissues from TCGA data. Differences in CDCA3 mRNA expression between tumors and unpaired normal tissues from TCGA and GTEx data were also analyzed. Then, we combined CDCA3 gene expression and clinical information to perform a univariate Cox regression analysis and plotted the corresponding forest plot through the “forestplot” R package to display the *p* value, HR, and 95% CI. Finally, to perform a reliable immune correlation assessment, we performed three different algorithms TIMER, xCell, and MCP-counter for the CDCA3 gene using the “immunedeconv” R package [26–28]. We extracted the expression information of SIGLEC15, IDO1, CD274, HAVCR2, PDCD1, CTLA4, LAG3, and PDCD1LG2 genes from the TCGA database. We then analyzed the correlation between CDCA3 gene expression and these immune checkpoint genes, and the above results were displayed as heatmaps.

### 2.2. Gene Expression Differential Analysis and Predictive Analysis

GEPIA is an interactive website for online analysis and mining of cancer data, designed by Zhang Zemin's Laboratory at the Peking University, mainly based on TCGA and GTEx database-related cancer data for analysis. It currently contains RNA expression profiling data for 9736 cancer and 8587 normal samples [29]. It can help medical researchers to carry out biomarker identification of related genes, expression profiling analysis of different cancer types or pathological stages, patient survival analysis, similar gene detection, correlation analysis, dimensionality reduction analysis, etc. In this study, based on the GEPIA website, we used a dichotomy to stratify cancer patients into two groups: CDCA3 high expression group and CDCA3 low expression group according to the expression of CDCA3 mRNA in cancer tissues. The association of CDCA3 expression with patient survival was analyzed using the Kaplan-Meier survival analysis. In addition, we have used a similar process in our multiple previous studies [30, 31].

### 2.3. Tumor Mutational Burden and Microsatellite Instability Analysis

With the development of molecular biology and next-generation sequencing technology, tumor mutational burden and microsatellite instability have become hotspots in cancer research. Therefore, we explored the correlation between tumor mutational burden, microsatellite instability, and CDCA3 gene expression. TMB is derived from Thorsson et al.'s 2018 article titled “The Immune Landscape of Cancer” [32]. MSI is derived from a 2017 article by Bonneville et al. entitled “Landscape of Microsatellite Instability Across 39 Cancer Types” [33]. Spearman's rank correlation coefficients were calculated to analyze the correlations of CDCA3 expression with the TMB and the MSI of each tumor sample.

### 2.4. Gene-Encoded Protein Interaction Network Analysis

The STRING database is a database developed by Peer Bork's team at the European Molecular Biology Laboratory that can be used to predict protein-protein interactions (https://string-db.org/) [34, 35]. It collects protein interaction information for many species, both experimentally validated and inferred by bioinformatic methods. This study explored the top 50 genes with the strongest correlation with CDCA3 through the STRING database and mapped the corresponding PPI network. Subsequently, we performed enrichment analysis for CDCA3-related gene sets using the online tools of the Metascape website (https://metascape.org/gp/index.html#/main/step1) [36] and further beautified them using Cytoscape software [37].

### 2.5. Gene Set Enrichment Analysis

Gene set enrichment analysis (GSEA) is a method for enrichment analysis of target genes, which can be used to detect the correlation between target genes and known functional gene sets. This study used the GTBA database to explore the relationship between the CDCA3 gene and the HALLMARK pathway (http://guotosky.vip:13838/GTBA/), and the results of the enrichment analysis were displayed using heatmaps and bar graphs. *p* < 0.05 was defined as a statistically significant difference.

### 2.6. Statistical Analysis

In this study, we used R software v4.0.3 for statistical analysis, used the Wilcoxon test to compare the expression differences of CDCA3 in the two groups of samples, and analyzed the corresponding data using statistical analysis software from multiple online databases. *p* < 0.05 was considered statistically significant.

## 3. Results

### 3.1. Transcriptional Level Analysis of CDCA3 in Pan-Cancer

To explore the expression of CDCA3 in pan-cancer, we first used the gene expression data in the TCGA database to compare the expression difference of CDCA3 in cancer and noncancer tissues and drew the corresponding violin plots. The results showed that CDCA3 was found in cancer tissues of BLCA, BRCA, CESC, CHOL, COAD, ESCA, GBM, HNSC, KIRC, KIRP, LIHC, LUAD, LUSC, PRAD, READ, SARC, STAD, and UCEC compared to normal tissues showing significantly high expression (Figures 1(a)–1(d)). Subsequently, due to the lack of data from normal tissues in the TCGA database, we combined the GTEx database to supplement data from more normal tissues. The results showed that compared with normal tissues, CDCA3 was found in ACC, BLCA, BRCA, CESC, CHOL, COAD, DLBC, ESCA, GBM, HNSC, KIRC, KIRP, LGG, LIHC, LUAD, LUSC, OV, PAAD, READ, SARC, SKCM, STAD, TGCT, UCEC, and UCS cancer tissues showing significantly high expression (Figures 1(e)–1(h)). Overall, CDCA3 is overexpressed dramatically in most cancer types and is likely to play a similar role as an oncogene in multiple cancer types.

### 3.2. Analysis of the Relationship between CDCA3 mRNA Levels and Different Clinicopathological Stages in Multiple Cancers

Cancer stage is a critical indicator for cancer patients. The higher the stage number, the more advanced the disease. Therefore, in this study, we investigated the expression of CDCA3 gene in different stages of various cancer types. The results showed that the expression of CDCA3 gene increased with the increase of stage in ACC, BRCA, KICH, KIRC, KIRP, LIHC, LUAD, and TGCT (Figures 2(a)–2(h)). This result suggests that CDCA3 may be positively correlated with the malignant progression of cancer.

### 3.3. Overall Survival Analysis of CDCA3 in Pan-Cancer

Overall survival (OS) was defined as the time from randomization to death from any cause. This indicator is often considered the best efficacy endpoint in oncology clinical trials. Therefore, in this study, we explored the OS of CDCA3 gene in pan-cancer. First, we obtained pan-cancer RNAseq data and corresponding clinical information from the TCGA database. We performed a univariate Cox regression analysis and displayed it using forest plots by the “forestplot” R package (Figure 3(a)). Subsequently, to test our previous results, we used the GEPIA database to explore the OS of CDCA3 gene in pan-cancer (Figure 3(b)). The results showed that high expression of CDCA3 gene was positively correlated with poor OS in ACC, KIRC, KIRP, LGG, LIHC, LUAD, MESO, PAAD, SARC, and SKCM patients (Figures 3(c)–3(l)).

### 3.4. Disease-Free Survival Analysis of CDCA3 in Pan-Cancer

Disease-free survival (DFS) is the time from randomization to disease recurrence or death due to disease progression. This indicator is often used as the primary endpoint of phase III clinical trials of antitumor drugs. Therefore, in this study, we explored the DFS of CDCA3 gene in pan-cancer. Similar to exploring OS in the previous step, we first performed a univariate Cox regression analysis and displayed it using a forest plot through the “forestplot” R package (Figure 4(a)). Subsequently, to test our previous results, we used the GEPIA database to explore the DFS of CDCA3 gene in pan-cancer (Figure 4(b)). The results showed that high expression of CDCA3 gene was positively correlated with poorer DFS in ACC, KIRC, KIRP, LGG, LIHC, LUAD, MESO, PCPG, PRAD, SARC, UCEC, and UVM patients (Figures 4(c)–4(n)).

### 3.5. Tumor Mutational Burden and Microsatellite Instability Analysis of CDCA3 in Pan-Cancer

TMB is highly correlated with the efficacy of PD-1/PD-L1 inhibitors, and most clinical studies using TMB as a marker have reached their endpoints with almost no failures. This allows some cancer patients to use TMB markers to predict immunotherapy's efficacy somewhat. MSI is caused by the functional defect of DNA mismatch repair in tumor tissue. The phenomenon of MSI accompanied by DNA mismatch repair deficiency is an important clinical tumor marker. Therefore, in this study, to further explore the role of CDCA3 in pan-cancer progression, we performed a Spearman correlation analysis of TMB/MSI for CDCA3 in pan-cancer. The first part of the results showed that CDCA3 was positively correlated between ACC, LUAD, STAD, BRCA, KICH, and TMB (Figure 5(a)). The second part of the results showed that CDCA3 was positively correlated between LUSC, UCEC, STAD, UCS, CHOL, and MSI (Figure 5(b)). This is helpful for a more comprehensive understanding of the biological significance of CDCA3 in pan-cancer.

### 3.6. Immune Correlation Analysis of CDCA3 in Pan-Cancer

To explore the correlation between CDCA3 and immune cell infiltration in pan-cancer, we used three algorithms TIMER, xCell, and MCP-counter to evaluate the correlation between CDCA3 expression in pan-cancer and immune cell infiltration in tumor tissue (Figures 6(a)–6(c)). The results showed that CDCA3 significantly correlated with various immune cell infiltrations in COAD, LUSC, STAD, and TGCT tissues. In contrast, CDCA3 is negatively associated with multiple immune cell infiltration in KIRC, LIHC, THCA, and THYM tissues. In addition, we further evaluated the correlation of CDCA3 with immune checkpoint gene expression in pan-cancer, and the results showed that CDCA3 expression was positively correlated with the expression of multiple immune checkpoint genes in THYM, TGCT, LUSC, and CESC, among which HAVCR2, PDCD1LG2, and SIGLEC15 genes were the most significant (Figure 6(d)).

### 3.7. Enrichment Analysis of CDCA3-Related Genes in Pan-Cancer

To perform enrichment analysis for CDCA3 genes, we performed enrichment analysis for CDCA3 and its closely related genes using STRING and Metascape databases. First, we used the STRING website to identify closely related genes interacting with CDCA3 (Figure 7(a)). To better analyze the functional mechanism between CDCA3 expression and human cancers, we performed an enrichment analysis using the Metascape database and obtained the two most important MCODE components from the analysis results. The two most important MCODE components are the regulation of mitotic cell cycle and the mitotic cell cycle process (Figure 7(b)). Next, we used the Metascape database to explore the underlying functional mechanisms of CDCA3 and its closely related genes. The top three biological effects were cell division, cell cycle, and mitotic cell cycle (Figures 7(c)–7(e)).

### 3.8. GSEA Analysis of CDCA3 in Pan-Cancer

Cancer researchers have increasingly used GSEA to assess the correlation between target genes and known phenotypic gene sets in recent years [30, 38, 39]. Therefore, in this study, we performed GSEA in the HALLMARK gene set targeting the CDCA3 gene in pan-cancer (Figures 8(a) and 8(b)). GSEA results indicated that CDCA3 genes were associated with abnormal activation of MYC TARGETS V2, MYC TARGETS V1, G2M CHECKPOINT, E2F TARGETS, and REACTIVE OXYGEN SPECIES PATHWAY. These data may provide a solid foundation for further studies of the CDCA3 gene and pave the way for future interventions.

## 4. Discussion

Despite the rapid development of molecular diagnostic and therapeutic strategies, there are currently no specific therapeutic targets for many types of cancer. Therefore, further research is urgently needed to discover more effective cancer biomarkers. Rapid cell growth and cell division are characteristic of nearly all cancer cells, and inappropriate expression of cell cycle regulatory proteins can contribute to cancer development [40, 41]. More and more studies have confirmed that dysregulated expression of CDCA3 plays a vital role in cancer progression. The clinical treatment effect of cancer patients with high expression of CDCA3 is worse, and CDCA3 may become a new potential prognostic marker and a new therapeutic target for cancer [42–45].

In this study, to gain an in-depth understanding of the differential expression of CDCA3 in pan-cancer, we first used the TCGA database to explore the mRNA expression level of CDCA3 in cancer tissues and normal tissues. There are different high expression degrees in more than ten types of cancers. However, while mining the TCGA database, we found that the sequencing results of normal tissues or paracancerous tissues included in the TCGA database are very scarce, which means that many cancer samples do not have the corresponding transcriptomes of normal tissues or paracancerous tissues, such as ACC, DLBC, LAML, LGG, MESO, OV, TGCT, and UCS. Therefore, in this study, we introduced the GTEx database, which contains more normal tissue expression information and combined it with the TCGA database to obtain more comprehensive transcriptome information. According to the mixed results of the TCGA and GTEx databases, the mRNA expression of CDCA3 was abnormally upregulated in almost all human cancers. Subsequently, we analyzed the potential prognostic value of CDCA3 in pan-cancer based on the GEPIA database. Our overall survival analysis results suggest that CDCA3 overexpression may be a predictive biomarker in multiple cancers, including ACC, KIRC, KIRP, LGG, LIHC, LUAD, MESO, PAAD, SARC, and SKCM. Compared with the corresponding normal samples, CDCA3 has different degrees of high expression in these cancer types. Patients with these cancer types in the high CDCA3 expression group had a poorer prognosis than those in the low CDCA3 expression group.

Several previous studies have shown that CDCA3 plays an essential role in the occurrence and development of cancer. Adams et al. used the GEO database, immunohistochemistry, and western blot methods to analyze the expression of CDCA3 in tumor and normal tissues of NSCLC, depleting CDCA3 with specific siRNA against three immortalized bronchial epithelial cell lines and seven NSCLC cell lines, to determine the biological function of CDCA3 in NSCLC [17]. In this study, Adams et al. also found that the CDCA3 protein was expressed in 81.1% of lung adenocarcinoma patients, and the expression rate in lung squamous cell carcinoma was as high as 61.9%. The expression of CDCA3 in NSCLC tumor tissue is significantly higher than that in normal tissue, and increased expression of CDCA3 is associated with a worse clinical prognosis [17]. Expression of CDCA3 was also elevated in NSCLC cell lines compared to immortalized bronchial epithelial cell lines. Reducing the expression of CDCA3 significantly reduced the proliferation of NSCLC tumor cells. CDCA3 depletion can cause poor cell cycle progression in the G2/M phase, upregulation of p21, and induction of cellular senescence. In addition, Uchida et al. used qRT-PCR and western blot to analyze the expression of CDCA3 mRNA and protein in oral squamous cell carcinoma cell lines and primary tumor tissues. And they used shRNA transfection technology to analyze the function of CDCA3 in vitro [46]. The results showed that the expression of CDCA3 at mRNA and protein levels was significantly increased in all tested cell lines and primary tumor tissues compared to normal cell lines and tissues. Compared with oral squamous cell carcinoma tissues, the protein expression level of CDCA3 in oral precancerous lesions was not significantly increased. Analysis of clinical data found that the expression level of CDCA3 was positively correlated with tumor size. In addition, using shRNA transfection technology to inhibit the expression of CDCA3 can arrest the cell cycle in the G1 phase and prevent cell proliferation. Uchida et al. showed that CDCA3 overexpression frequently occurs in oral squamous cell carcinoma, which is closely related to the development of oral squamous cell carcinoma [46].

In additional studies, Phan et al. found that CDCA3 mRNA expression in breast cancer tissues was significantly higher than that in normal controls using bioinformatics analysis and was associated with the overall survival of patients [16]. CDCA3 mRNA expression was significantly upregulated in gastric cancer tissues compared with normal tissues [18, 24]. The study by Qian et al. revealed that CDCA3 mRNA expression was significantly upregulated in colorectal cancer tissues and correlated significantly with tumor size, TNM stage, and lymph node invasion [19]. Mechanistic analysis showed that CDCA3 could affect the expression of downstream molecule p21 by regulating the transcription factor E2F1, thereby affecting the G1/S transition of the cell cycle. CDCA3 can also promote the proliferation of colorectal cancer cells by activating the NF-*κ*B/cyclin D1 pathway [25]. Qian et al. knocked out the CDCA3 gene in the colon cancer cell line SW480, significantly reducing cell proliferation [19]. Chen et al. found that HoxB3 can promote prostate cancer progression by upregulating the expression of CDCA3, and blocking this pathway may be a potential therapeutic strategy for prostate cancer [23]. The study by Bi et al. pointed out that the CDCA3-related path is expected to become a new molecular strategy for leukemia treatment [21]. Zhang et al. knocked out the CDCA3 gene in gastric cancer cells, which inhibited cell proliferation and induced G0/G1 phase arrest [18]. The expression level of CDCA3 can be regulated by transcription and protein degradation in the G1 phase [47, 48]. In addition, Hu et al. found that CDCA3 may cooperate with OY-TES-1 to participate in the proliferation, migration, invasion, and apoptosis of liver cancer cells [49]. Li et al. found that low expression of CDCA3 was associated with better overall survival in bladder cancer patients [20].

In addition, our study still has some limitations, such as the lack of clinical and laboratory data. Therefore, in the future, we will further explore the predictive value and biological role of CDCA3 in clinicopathological samples and cancer cell experiments.

## 5. Conclusions

Taken together, CDCA3 is a trigger for mitotic entry and is involved in regulating the initiation and termination of cellular mitosis. Whether in our study or in previous studies, CDCA3 is abnormally high expressed in various types of cancer and has a close relationship with the occurrence, development, and prognosis of cancer. CDCA3 can promote cancer cell proliferation and reduce the survival rate of cancer patients. It can be used as a prognostic indicator of cancer and is expected to become a new target for cancer therapy. Currently, the research on CDCA3 is immature, and more biological functions and mechanisms remain to be revealed.

## Figures and Tables

**Figure 1:** Expression distribution of CDCA3 in pan-cancer. (a–d) Violin plots show the expression distribution of CDCA3 gene in various tumor tissues and normal tissues based on the TCGA database. (e–h) Combining TCGA and GTEx databases, violin plots show the expression distribution of CDCA3 gene in various tumor tissues and normal tissues. The abscissa represents different tumor tissues, the ordinate represents the gene expression distribution, red represents the tumor group, and blue represents the normal group. ^∗^*p* < 0.05, ^∗∗^*p* < 0.01, and ^∗∗∗^*p* < 0.001.

**Figure 2:** Violin plots show the expression of CDCA3 in different stages of various tumors. (a) ACC, (b) BRCA, (c) KICH, (d) KIRC, (e) KIRP, (f) LIHC, (g) LUAD, and (h) TGCT.

**Figure 3:** OS analysis of CDCA3 in pan-cancer. (a) The forest plot shows the univariate Cox analysis of CDCA3 gene in OS of various tumor patients, including *p* value, risk coefficient HR, and confidence interval. (b) Heatmap showing OS of CDCA3 gene in pan-cancer. (c–l) Kaplan-Meier curves show OS of CDCA3 gene in ACC, KIRC, KIRP, LGG, LIHC, LUAD, MESO, PAAD, SARC, and SKCM.

**Figure 4:** DFS analysis of CDCA3 in pan-cancer. (a) The forest plot shows the univariate Cox analysis of CDCA3 gene in DFS of various tumor patients, including *p* value, risk coefficient HR, and confidence interval. (b) Heatmap showing DFS of CDCA3 gene in pan-cancer. (c–n) Kaplan-Meier curves show DFS of CDCA3 gene in ACC, KIRC, KIRP, LGG, LIHC, LUAD, MESO, PCPG, PRAD, SARC, UCEC, and UVM.

**Figure 5:** Mutational analysis of CDCA3 in pan-cancer. (a) Spearman correlation analysis of CDCA3 gene expression and TMB. (b) Spearman correlation analysis of CDCA3 gene expression and MSI. The size of the dots represents the size of the correlation coefficient, and the different colors represent the significance of the *p* value. The bluer the color, the smaller the *p* value.

**Figure 6:** Immune correlation analysis of CDCA3 in pan-cancer. (a–c) Based on three different algorithms, TIMER, xCell and MCP-counter, the heatmap shows the correlation between CDCA3 expression and immune cell infiltration in pan-cancer. (d) Heatmap showing the correlation results between CDCA3 expression in pan-cancer and immune checkpoints. These immune checkpoints are SIGLEC15, IDO1, CD274, HAVCR2, PDCD1, CTLA4, LAG3, and PDCD1LG2.

**Figure 7:** Enrichment analysis of CDCA3-related genes in pan-cancer. (a and b) Protein-protein interaction network and MCODE components are identified in CDCA3-related genes. (c) Bar graph of enriched terms across CDCA3-related genes, colored by *p* values. (d) Network plot showing enriched terms in CDCA3-related genes colored by cluster-ID. (e) Network plot showing enriched terms in CDCA3-related genes colored by *p* value.

**Figure 8:** GSEA analysis of CDCA3 in pan-cancer. (a and b) Heatmap and bar graph showing the results of GSEA of CDCA3 gene in pan-cancer. Notably, purple represents activation, and green represents inhibition. ^∗^*p* < 0.05 and ^∗∗^*p* < 0.01.

## Data Availability

The data used to support the findings of this study are available from the corresponding author upon request.

## Abbreviations

CDCA3: Cell division cycle-associated protein 3
TCGA: The Cancer Genome Atlas
GTEx: Genotype-tissue expression
GEPIA: Gene expression profiling interactive analysis
TIMER: Tumor immune estimation resource
GSEA: Gene set enrichment analysis
SIGLEC15: Sialic acid binding Ig like lectin 15
IDO1: Indoleamine 2,3-dioxygenase 1
CD274: CD274 molecule
HAVCR2: Hepatitis a virus cellular receptor 2
PDCD1: Programmed cell death 1
CTLA4: Cytotoxic T-lymphocyte associated protein 4
LAG3: Lymphocyte activating 3
PDCD1LG2: Programmed cell death 1 ligand 2
ACC: Adrenocortical carcinoma
BLCA: Bladder urothelial carcinoma
BRCA: Breast invasive carcinoma
CESC: Cervical squamous cell carcinoma and endocervical adenocarcinoma
CHOL: Cholangiocarcinoma
COAD: Colon adenocarcinoma
DLBC: Lymphoid neoplasm diffuse large B-cell lymphoma
ESCA: Esophageal carcinoma
GBM: Glioblastoma multiforme
HNSC: Head and neck squamous cell carcinoma
KIRC: Kidney renal clear cell carcinoma
KIRP: Kidney renal papillary cell carcinoma
LGG: Brain lower grade glioma
LIHC: Liver hepatocellular carcinoma
LUAD: Lung adenocarcinoma
LUSC: Lung squamous cell carcinoma
OV: Ovarian serous cystadenocarcinoma
PAAD: Pancreatic adenocarcinoma
READ: Rectum adenocarcinoma
SARC: Sarcoma
SKCM: Skin cutaneous melanoma
STAD: Stomach adenocarcinoma
TGCT: Testicular germ cell tumors
UCEC: Uterine corpus endometrial carcinoma
UCS: Uterine carcinosarcoma.
